# In-hospital cerebrovascular complications following orthotopic liver transplantation: A retrospective study

**DOI:** 10.1186/1471-2377-8-52

**Published:** 2008-12-22

**Authors:** Li Ling, Xiaoshun He, Jinsheng Zeng, Zhijian Liang

**Affiliations:** 1 Department of Neurology and Stroke Centre, First Affiliated Hospital, Sun Yat-Sen University, No. 58 Zhongshan Road 2, Guangzhou, 510080, PR China; 2 Department of Organ Transplantation, First Affiliated Hospital, Sun Yat-Sen University, No. 58 Zhongshan Road 2, Guangzhou, 510080, PR China; 3 Department of Neurology and Stroke Centre, First Affiliated Hospital, Guangxi Medical University, No. 23, Shuangyong Road, Nanning, 530021, PR China

## Abstract

**Background:**

Cerebrovascular complications are severe events following orthotopic liver transplantation (OLT). This study aimed to observe the clinical and neuroimaging features and possible risk factors of in-hospital cerebrovascular complications in the patients who underwent OLT.

**Patients and methods:**

We retrospectively reviewed 337 consecutive patients who underwent 358 OLTs. Cerebrovascular complications were determined by clinical and neuroimaging manifestations, and the possible risk factors were analyzed in the patients with intracranial hemorrhage.

**Results:**

Ten of 337 (3.0%) patients developed in-hospital cerebrovascular complications (8 cases experienced intracranial hemorrhage and 2 cases had cerebral infarction), and 6 of them died. The clinical presentations were similar to common stroke, but with rapid deterioration at early stage. The hematomas on brain CT scan were massive, irregular, multifocal and diffuse, and most of them were located at brain lobes and might enlarge or rebleed. Infarcts presented lacunar and multifocal lesions in basal gangliar but with possible hemorrhagic transformation. The patients with intracranial hemorrhage had older age and a more frequency of systemic infection than non-intracranial hemorrhage patients. (P = 0.011 and 0.029, respectively).

**Conclusion:**

Posttransplant cerebrovascular complications have severe impact on outcome of the patients who received OLT. Older age and systemic infection may be the possible risk factors of in-hospital intracranial hemorrhage following OLT.

## Background

With the rapid development of transplant technique and immunosuppressive therapy, orthotopic liver transplantation (OLT) has been carried out all over the world and accepted as one of the most effective treatments for the patients with end-stage liver diseases. However, postoperative complications are still the most important causes resulting in death of patients undergoing OLT. The incidences of posttransplant cerebrovascular complications or intracranial hemorrhage were 2.2%–3.9% in United States [1-3], 3.3% in United Kingdom[4], 3.7% in Chile[5], 6% in Spain[6], 6.5% in Hong Kong[7] clinically, and 32.7% in post-mortem patients after OLT in United States[8]. But cerebrovascular complications following OLT in patients of mainland China have not been reported. In the present study, we reported the incidence, mortality and clinical and neuroimaging features, then analyzed the possible risk factors of in-hospital cerebrovascular complications in patients following OLT at a center in southern China.

## Methods

### Patients

We retrospectively reviewed 337 consecutive patients who underwent 358 OLTs in which 19 patients had a second transplant, and one had a third transplant, at an organ transplant center in southern China from Janurary 1st,1996 to June 30th, 2005. The mean age was 47 ± 11.5 years (3 months to 75 years), and 288 of 337 patients were males. The primary liver diseases before OLT are listed in Table 1.

**Table 1:** The primary liver diseases before orthotopic liver transplantation

The primary liver diseases	Cases (%)
Primary hepatic carcinoma	198 (58.75%)
Cirrhosis	94 (27.89%)
Hepatitis B	21 (8.01%)
Secondary hepatic carcinoma	6 (1.78%)
Polycystic liver disease	4 (1.19%)
Giant hemangioma of the liver	3 (0.89%)
Primary sclerosing cholangitis	3 (0.89%)
Drug-induced hepatitis	2 (0.59%)
Congenital biliary atresia	2 (0.59%)
Hepatitis C	1 (0. 30%)
Congenital hepatic fibrosis	1 (0. 30%)
Budd-Chiari syndrome	1 (0. 30%)
Acute fatty liver and liver function failure of pregnancy	1 (0. 30%)
Total	337 (100%)

### Management

All patients underwent OLT using Piggyback technique and were managed in an intensive care unit before being transferred to a general ward following surgery. FK506, cyclosporine A or corticosteroids were used as immunosuppressives and their serum level was measured daily postoperativly. Blood tests such as blood platelet counts, prothrombin time (PT), activated partial prothrombin time (APPT), the function of the liver and kidney and other necessary tests were measured routinely. Brain computed tomography (CT) or magnetic resonance imaging (MRI) was performed in patients when neurological symptoms occurred after OLT.

We focused on the clinical and neuroimaging features of the patients with in-hospital cerebrovascular complications following OLT, and analyzed the possible risk factors in the patients with intracranial hemorrhage.

The research protocol was approved by the local ethical committee for clinical research and all procedures involving the participant were conducted according to institutional guidelines in compliance with the regulations. Both oral and written informed consents were obtained from the patients or their families.

### Statistical analysis

All statistical calculations were performed on microcomputer using SPSS13.0 (SPSS Inc). Continuous variables were compared using two tails student's t-test, and categorical variables analyzed by a chisquare analysis or Fisher's exact test. A *p *value less than 0.05 was considered significantly.

## Results

In all 10 patients (6 males, 4 females) aged 56 ± 8.4 years (40 to 67 years) developed in-hospital cerebrovascular complications following OLT, resulting in an incidence of 3.0% in 337 patients. The mean in-hospital time were 39 ± 21.7 days (8 to 70 days). All patients with cerebrovascular complications had brain CT scan. Among them, eight patients (8/337, 2.4%) experienced intracranial hemorrhage, including 5 with lobe hematomas, 2 with subdural hematomas, and 1 with lobe and subarachnoid hemorrhage, and 7 of 8 intracranial hemorrhages occurred within posttransplant 1 month. The clinical presentations, such as unconsciousness, headache, aphasia, hemiparesis, seizures, were similar to common hemorrhagic stroke, but with rapid deterioration at early stage. Five of 8 patients with intracranial hemorrhage deteriorated clinically and then died within two weeks after onset, including two patients with enlargement of hematoma and intraventricular mass, and a marked midline shift on repeated CT. Two of 337 (0.6%) patients had lacunar cerebral infarctions on the 6th and the 58th postoperative day respectively. One patient's lesions located in basal ganglia and cerebellum, the other patient with generalized seizures at the oneset had a lacunar infarction at left basal ganglia. Although the seizure stopped soon after antiepileptic therapy, the aptient became apathia and reactiveless, then persistent coma. Neurological examination showed bilateral unclear papilla opticas with left papilla optica retinal vein bleeding and stiff neck. It's a pity that the repeat CT scan was not done due to the severe conditions. The patient died of multiple organ failure on the 11th days after OLT. All clinical and laboratory data, as well as brain CT findings of patients with cerebrovascular complications following OLT are shown in an Additional Table (see additional file 1).

Among the 8 patients with intracranial hemorrhage, two of them received decompressive craniectomy and evacuation of intracranial hematoma, but both died of brain herniation soon after the surgery. Other 6 patients received medical treatement, and 3 of them survived. One of 2 patients with cerebral infarction died. Altogether, six of 10 patients with in-hospital cerebrovascular complications died following OLT.

To analyze the possible risk factors and outcome of intracranial hemorrhage following OLT, we compared the clinical and laboratory data between the patients with and without intracranial hemorrhage (Table 2). In our series, the patients with intracranial hemorrhage had older age and a more frequency of systemic infection than non-intracranial hemorrhage patients (56.3 ± 8.7 vs 46.7 ± 11.7 years old,*p *= 0.011; 7/8 vs152/329, *p *= 0.029, respectively). The patients over 55 years were prone to have intracranial hemorrhage than those less than 55 years (5/75 vs 3/262, *p *= 0.015). Additionly, seven of 8 patients with systemic bacterial or fungal infection experienced intracranial hemorrhage, which had a more frequency than those without infection (7/155 vs 1/182, *p *= 0.026). The patients over 55 years with systemic infection had more frequency of intracranial hemorrhage than those less than 55 years and without systemic infection (5/37 vs 1/52,*p *= 0.043). Seven of 8 patients with intracranial hemorrhage had infection, including 4 patients experienced bacterial pneumonia, one had an aspergillus pneumonia, an aspergillus combinded Candida tropicalis pneumonia and a bacterial pneumonia combinded urinary tract infection respectively. The patients with intracranial hemorrhage had a higher mortality rate than those without intracranial hemorrhage (5/8 vs 74/329, *p *= 0.019).

**Table 2:** Comparison of clincal features between the patients with and without intracranial hemorrhage after orthotopic liver transplantation

Features	intracranial hemorrhage (n = 8)	non-intracranial hemorrhage (n = 329)
age (years)	56.3 ± 8.7 (40–67)	46.7 ± 11.7 (0.3–75)*
>55 years	5 (62.5%)	70 (21.3%)
≤55 years	3 (37.5%)	259 (78.7%)
operative time (h)	6.3 ± 0.5 (5.5–10.0)	7.2 ± 1.9 (4–15)
previous abdominal surgery	4 (50%)	113 (34.3%)
retranplatation	0 (0)	20 (6.1%)
introperative blood loss volume (ml)	4312.5 ± 4566.5 (1500–15000)	3900.0 ± 4389.7 (100–38000)
thrombocytopenia	1 (12.5%)	66 (20.1%)
PT(s)	16.3 ± 5.2 (9.8–22.6)	18.8 ± 6.4 (9.7–46.3)
APTT(s)	35.7 ± 11.4 (26.1–58.6)	39.2 ± 13.6 (22.9–180)
preoperative hypertension	0 (0)	5 (1.5%)
introperative hypotension	5 (62.5%)	110 (33.4%)
postoperative hypertension	2 (25%)	23 (7.0%)
bacterial or fungal infections	7 (87.5%)	148 (45.0%)*
sepsis	1 (12.5%)	29 (8.8%)
bleeding at extracerebral sites	1 (12.5%)	31 (9.4%)
death	5 (62.5%)	74 (22.5%)*

*: vs intracranial hemorrhage, *p *< 0.05. PT: prothrombin time; APTT: activated partial prothrombin time.

## Discussion

### Incidence and mortality rate

In the past 20 years, more and more patients with various end-stage diseases have benefited from organ transplantation. But cerebrovascular events, especially intracranial hemorrhage, have been concerned as severe neurological complications after transplantation. The reported clinical incidences of cerebrovascular complications were 1.7%–6.5% [1-7], and the mortality rate of cerebrovascular complications or intracranial hemorrhage were 57%–100% following OLT[1,3,7]. Moreover, the incidence was 32.7% in autopsy cases of patients who underwent OLT[8]. Cerebrovascular complications are also common in other transplantation patients. It has been reported that the incidence of ischemic and hemorrhagic strokes was 6.8% after kidney transplantation[9], 2.9% after bone marrow transplantation[10], 0.9% after reduced-intensity stem cell transplantation[11] and 2% in pediatric patients after cardiac transplantation[12]. Our study showed that the incidence of cerebrovascular complications in patients of southern China who underwent OLT was 3.0%, and 6 of 10 died, which was similar to the previous international reports [1-7]. These data indicate cerebrovascular events, especially intracranial hemorrhage, are severe posttransplant complications which deserve more attention for the neurologists, neuro-intensivists and surgeons for organ transplantion, and more endeavours should be done prospectively to identify or aviod such complications in clinical practice.

### Clinical and neuroimaging features

In our study, the intracranial hemorrhage patients presented with unconsciousness, headache, aphasia, hemiparesis, seizures, which was consistent with the findings of previous report[2]. These presentations were similar to common stroke, but with more urgent onset, progressing clinical course and rapid deterioration at early stage. In our experience, sudden conscious disturbance (or loss of consciousness) after OLT was strongly associated with intracranial hemorrhage. In the present of coagulopathy, metabolic disturbance or multiple organ failure in early postoperative time, liver transplantation recipients were prone to developed massive intracranial hematomas. Moreover, these hematomas were not prone to cease spontaneously and might enlarge gradually or rebleed, even with a tendency to form cerebral herniation, which results in the death. It is important to examine the consciousness and pupils in patients after OLT. Brain CT scan shoud be performed promptly to identify whether intracranial hemorrhage occurs once the patient has sudden conscious disturbance or loss of consciousness following OLT. Additionally, liver transplantation recipients may occurr ischemic infarction due to the haemodynamic change and coagulopathy, and then develop hemorrhagic infarction, then deteriorated rapidly.

### Possible risk factors

Most liver transplantation recipients are in the end-stage of liver diseases, preoperative liver dysfunction even liver failure results in thrombocytopenia and absence of coagulation factors. Moreover, liver function may not return to normal level in the postoperative early stage. All these could result in coagulopathy, which can trigger intracranial hemorrhage after OLT[2]. But in our series, no significant differences were found in the incidence of thrombocytopenia, PT, or APPT between the patients with and without intracranial hemorrhage, which suggests that the causes of intracranial hemorrhage after OLT are multiple and complex, except for coagulopathy, there may be other factors responsible for this complication. In our study, we found that intracranial hemorrhage patients were older than non-intracranial hemorrhage patients, moreover, the patients over 55 years had a more frequency of intracranial hemorrhage than those less than 55 years old. Additionly, the patients with systemic infection had a more frequency of intracranial hemorrhage than those without infection. The results indicate that older age and systemic infection might be important risk factors of intracranial hemorrhage following OLT. Cox and colleagues[13] reported that an 11-year-old boy who had cystic fibrosis died of an intraventricular and intracerebral hemorrhage caused by an aspergillus brain abscess on the 48th day after OLT. Wijdicks and colleagues[2] reported that in the group of 8 patients with intracranial hemorrhage after OLT, one had a Candida-associated mycotic aneurysm demonstrated by autopsy and another had disseminated aspergillosis. Generally, it is presumed that under the condition of systemic infection related to immunosuppresion following OLT, aspergillus, toxoplasma and any virulent bacterial organism may lead to inflammation of the arterial wall and formation of an aneurysm[2,14-16]. In our series, seven of the 8 patients with intracranial hemorrhage had systemic bacterial or fungal infection, and all that them had pneumonia, including 4 with bacterial pneumonia, one with aspergillus pneumonia, one with aspergillus combinded Candida tropicalis pneumonia and one with bacterial pneumonia combinded urinary tract infection respectively. But it was very pitiful that no evidence to support bacterial or fungal infection is the direct cause of intracranial hemorrhage due to no vascular image or post-mortem exams in the present study. A published study showed that patients with introperative hypotension were prone to develop cerebral infarction after OLT[7]. In the present study, one patient over 60 years old with cerebral infarction indeed had introperative hypotension, indicating introperative hypotension may be a potential risk factor of cerebral infarction after OLT.

## Conclusion

Although posttransplant cerebrovascular complications are not common, they have severe impact on outcome of the patients who received OLT. Age and systemic infection may be the possible risk factors of in-hospital intracranial hemorrhage following OLT. More effctive measures should be taken to prevent posttransplant infection, such as improvement of patient's systemic condition, bacteriologic surveillance and infection control measures. It is urgent to early diagnosis and take more prompt systemic antibiotic/antifungal therapy once infection occurs, especially in old patients. Further prospective study is necessary to explore the risk factors and optimize the preventive and therapeutic regimen of intracranial hemorrhage following OLT.

## Competing interests

The authors declare that they have no competing interests.

## Authors' contributions

LL collected the data and wrote the primary manuscript. HX participated in the study. ZJ designed the study, interpreted the results and critically revised the manuscript. LZ assisted with the statistical analysis. All authors read and approved the final manuscript.

## Pre-publication history

The pre-publication history for this paper can be accessed here:



## Supplementary Material

Additional file 1 **All clinical and laboratory data, as well as brain CT findings of patients with cerebrovascular complications following orthotopic liver transplantation are shown this additional table.** Click here for file
